The article "Paeoniflorin alleviates NG-nitro-L-arginine methyl ester (L-NAME)-induced gestational hypertension and upregulates silent information regulator 2 related enzyme 1 (SIRT1) to reduce H2O2-induced endothelial cell damage" was published in 2022. Journal: Bioengineered.

# Paeoniflorin alleviates NG-nitro-L-arginine methyl ester (L-NAME)-induced gestational hypertension and upregulates silent information regulator 2 related enzyme 1 (SIRT1) to reduce H_2_O_2_-induced endothelial cell damage

**DOI:** 10.1080/21655979.2021.2024325

**Published:** 2022-01-14

**Authors:** Jingjing Wu, Dongmei Zhang, Linlin Hu, Xiaowei Zheng, Caihong Chen

**Affiliations:** a Department of Obstetrics, The Second Affiliated Hospital of Fujian Medical University, Quanzhou, Fujian, P.R. China; b Clinical Laboratory, The Second Affiliated Hospital of Fujian Medical University, Quanzhou, Fujian, P.R. China

**Keywords:** Paeoniflorin, pregnancy hypertension, SIRT1, vascular endothelial cell dysfunction

## Abstract

Pregnancy-induced hypertension (PIH) is a leading cause of maternal mortality. Paeoniflorin has been reported to alleviate hypertension, thus relieving the injury of target organ. This study aimed to investigate the role of paeoniflorin in PIH development by regulating SIRT1 in rats. The mean arterial pressure (MAP), urine protein and histopathological damage of placenta in gestational hypertension rats were, respectively, detected by noninvasive tail-artery pressure measuring instrument, BCA method and H&E staining. The viability of human umbilical vein endothelial cells (HUVECs) treated with paeoniflorin or/and H_2_O_2_ was observed by CCK-8 assay. SIRT1 protein expression in HUVECs treated with paeoniflorin or/and H_2_O_2_ was analyzed by Western blot. Tunel assay, wound healing assay and tube formation assay were used to detect the apoptosis, migration and tube formation of HUVECs administrated with paeoniflorin or/and H_2_O_2_ or/and EX527 (SIRT1 inhibitor). As a result, MAP, urine protein and histopathological damage of placenta were enhanced in PIH rats, which were then alleviated by paeoniflorin. Paeoniflorin decreased the levels of sFlt-1, PlGF and VEGF in serum and placental tissues of gestational hypertension rats as well as the inflammatory response and oxidative stress. In addition, paeoniflorin promoted the expressions of SIRT1 and NO/eNOS and inhibited the production of iNOS in gestational hypertension rats to improve vascular endothelial cell injury. However, SIRT1 inhibition could suppress the protective effects of paeoniflorin on endothelial dysfunction of H_2_O_2_-induced HUVECs. In conclusion, paeoniflorin could improve gestational hypertension development by upregulating SIRT1.

## Introduction

Pregnancy-induced hypertension (PIH, gestational hypertension) is a systemic disease, which especially occurs in pregnant women after 20 weeks of gestation. Hypertension and proteinuria are main clinical manifestations. If the disease is not controlled in time, it will seriously affect the life safety and quality of life of pregnant women as well as their fetuses [1]. It is defined as systolic blood pressure (SBP) >140 mmHg and diastolic blood pressure (DBP) >90 mmHg [2]. Gestational hypertension is considered to be one of the leading causes of maternal death during pregnancy, accounting for approximately 14% of maternal deaths worldwide [3].

Paeoniflorin is the main component of total glycosides of Paeonia lactiflora, which is derived from Chinese herbal medicines such as peony root and purple peony root [4]. Modern pharmacological studies have found that total glucosides of Paeonia lactiflora have the effects of relieving pain, alleviating inflammatory response, protecting liver, and inhibiting autoimmune reaction through multiple ways [5]. Paeoniflorin improves chronic hypoxia/SU5416-induced pulmonary arterial hypertension by inhibiting the transformation of endothelial cells to mesenchymal cells [6]. Paeoniflorin, benzoylpaeoniflorin, mudanpioside C and paeonol effectively block Ca^2+^ channels under the action of voltage, thus exserting calcium antagonism [7]. Paeoniflorin decreases blood pressure to improve cardiac remodeling by inhibiting MAPK signaling pathway in spontaneously hypertensive rats (SHR) [8]. The combination of paeoniflorin and metoprolol improves microcirculation, upregulates eNOS expression, and alleviates endothelial dysfunction in SHR [9]. Paeoniflorin can obviously decrease blood pressure variability, stabilize blood pressure, and alleviate organ damage in SHR [10]. However, the role of paeoniflorin in alleviating PIH remains unknown.

In recent years, it has been found that the deacetylase silent information regulator 2 related enzyme 1 (SIRT1) plays an important role in the functional regulation of peripheral circulatory system [11]. SIRT1 decreases the levels of HMGB1 and HSP70 released from IL-6 induced human umbilical vein endothelial cells (HUVECs) and preeclampsia patient serum [12]. Paeoniflorin inhibits the apoptosis of ox-low density lipoprotein-induced HUVECs and the expressions of adhesion molecules by upregulating SIRT1, thereby alleviating ox-low density lipoprotein-induced HUVEC injury [13].

Therefore, whether and how paeoniflorin exerts its protective effects on gestational hypertension needs to be explored. The present study first explored the effects of paeoniflorin on the L-NAME-induced gestational hypertension rat model, followed by the H2O2-induced HUVEC model to further explore the mechanism of protective effects of paeoniflorin on endothelial cell dysfunction.

## Materials and methods

### Gestational hypertension rat model and paeoniflorin treatment

Wistar rats (20 females, 10 males; 10–12 weeks old; 180–220 g) were obtained from Shanghai Jiesijie Experimental Animal Co., Ltd. The rats were housed in a room with controlled temperature (23 ± 2°C), humidity (55 ± 5%) and artificial 12-h light/dark cycle, and were permitted to eat as much food and tap water as they wanted. All protocols were approved by the Animal Care and Research Committee of the Second Affiliated Hospital of Fujian Medical University.

The estrous female and male mice were caged together at 2:1 overnight, and sperm was found by microscopic examination of vaginal saline rinse solution of female mice on the next day, which was considered as day 1 of gestation (D1). A total of 20 female pregnant rats were randomly divided into four groups: Control pregnant rats (Control group), gestational hypertension rats (PIH group), PIH rats + paeoniflorin (100 mg/kg) [PIH + Pae (100 mg/kg) group] and PIH rats + paeoniflorin (300 mg/kg) [PIH + Pae (300 mg/kg) group]. Nitric oxide synthase inhibitor NG-nitro-L-arginine methylester (L-NAME; 250 mg/kg/d) was administered by intraperitoneal injection from day 11 to day 18 of gestation (D11-D18) to induce gestational hypertension rats. Control group was injected with the same amount of normal saline. Paeoniflorin was administered with gastric infusion from day 2 to day 19 of gestation (D2-D19).

### Blood pressure measurement

Systolic blood pressure (SBP) and diastolic blood pressure (DBP) in pregnant rats were measured at day 8 and day 18 of gestation using BP-2000 Series II noninvasive tail-artery pressure measuring instrument (Visitech Systems, Apex, NC, USA) to calculate the mean arterial pressure (MAP).

### Bicinchoninic acid (BCA) method

On day 9 and day 19 of gestation, rats were chosen by the random selection mechanism and transferred to metabolic cages to collect urine for 24 h. Urine protein concentration was measured using the BCA method.

### Hematoxylin and eosin (H&E) staining

On day 19 of gestation, rats were euthanized with 2% sodium pentobarbital (200 mg/kg) by intraperitoneal injection to obtain placental tissues. Placental tissues were fixed with 4% formalin at room temperature for 24 h and paraffin-embedded, which were then cut into 5 µm-thick sections. Tissue sections were stained with H&E at room temperature for 1–2 min and observed under a light microscope.

### Enzyme-linked immunosorbent assay (ELISA)

The concentrations of soluble fms-like tyrosine kinase-1 (sFlt-1), placental growth factor (PlGF) and vascular endothelial growth factor (VEGF) in serum, concentrations of TNF-α, IL-6, IL-1β and MCP-1 in serum and placental tissues as well as concentrations of MDA, SOD and GSH-Px in placental tissues were measured using Rat sFlt-1 ELISA Kit (cat. no. JL48077; Jonln), Rat PlGF ELISA Kit (cat. no. JL11559; Jonln), Rat VEGF ELISA Kit (cat. no. PV960; Beyotime), Rat TNF-α ELISA Kit (cat. no. PT516; Beyotime), Rat IL-6 ELISA Kit (cat. no. PI328; Beyotime), Rat IL-1β ELISA Kit (cat. no. PI303; Beyotime), Rat MCP-1 ELISA Kit (cat. no. RAB0058-1KT; Merck), MDA Assay Kit (cat. no. ab238537; Abcam), SOD (cat. no. CS0009-1KT; Merck) and GSH-Px Assay Kit (cat. no. E-BC-K096-M; Elabscience) according to the manufacturer’s directions.

### Reverse transcription quantitative PCR

The total RNA was extracted from placental tissues using TRIzol® reagent, and 1 μg total RNA was converted to cDNA using PrimeScript™ RT reagent kit. Quantitative PCR was performed using SYBR Green Premix Ex Taq. The mRNA expression of targeted genes was calculated using 2^−ΔΔCq^ method [14]. The primers used were as follows: sFlt-1 forward, 5ʹ-GATGGGTTACCTGCGACTG-3ʹ and reverse, 5ʹ-CCGGGTCTGGAAACGATG-3ʹ; PlGF forward, 5ʹ-TCAGAGGTGGAAGTGGTA-3ʹ and reverse, 5ʹ-ACACAGTGCAGATTCTCA-3ʹ; VEGF forward, 5ʹ-ACCATGAACTTTCTGCTC-3ʹ and reverse, 5ʹ-GGACGGCTTGAAGATATA-3ʹ; GAPDH forward, 5ʹ-AGTGCCAGCCT-CGTCTCATA-3ʹ and reverse, 5ʹ-TGAACTTGCCGTGGGTAGAG-3ʹ.

### Cell culture

HUVECs (PCS-100-013™) were bought from ATCC (Manassas) and cultured in M199 medium (Gibco) added with 10% fetal bovine serum (FBS), 10 mM HEPES (Sigma Aldrich) and 1% penicillin/streptomycin solution.

### Western blot

Tissue lysates and cell lysates were prepared using RIPA buffer (Solarbio, China) to obtain total proteins. Proteins (50 µg) were separated on SDS-PAGE and transferred on polyvinylidene fluoride (PVDF) membranes (Millipore, USA). The membranes were blocked with 5% (w/v) skimmed milk solution for 1 h, and incubated with rabbit primary antibodies (Abcam) against sFlt-1, PlGF, SIRT1, eNOS and GAPDH at 4°C for 12 h. Next, the membranes were washed and incubated with appropriate anti-rabbit HRP-conjugated secondary antibodies at 37°C for 1 h. Protein bands were detected using chemiluminescence and band intensities were analyzed using Quantity One software 4.6.2 (Bio-Rad, Hercules, CA, USA).

### Measurement of NO and iNOS

The expression levels of NO and iNOS in serum and culture supernatant of HUVECs were measured using Total NO Assay Kit (cat. no. S0023; Beyotime) and Rat iNOS ELISA Kit (cat. no. JL21441; Jonln) according to the manufacturer’s directions.

### CCK-8 assay

One experiment was that HUVECs were seeded in a 96-well microplate at a density of 5 × 10^3^ cells/well, and then treated with different concentrations of paeoniflorin (50, 100 and 200 μM) for 24 h. Then, CCK-8 solution (10 μL/well) was put into the wells to incubate the cells at 37°C for 1.5 h. Another experiment was that HUVECs were seeded in a 96-well microplate at a density of 5 × 10^3^ cells/well, and then exposed to H_2_O_2_ for 2 h. After H_2_O_2_ induction, HUVECs were further treated with different concentrations of paeoniflorin (50, 100 and 200 μM) for 24 h. Subsequently, CCK-8 solution (10 μL/well) was put into the wells to incubate the cells at 37°C for 1.5 h. The absorbance values (cell viability) were recoded with a microplate reader at a wavelength of 490 nm.

### TUNEL assay

Briefly, HUVECs that induced by H_2_O_2_ or/and treated with paeoniflorin or/and treated with EX527 (SIRT1 inhibitor) were cultured at 37°C for 24 h. Then, cells were fixed in 4% paraformaldehyde for 30 min, treated with proteinase K (20 μg/ml) for 20 min, and incubated with terminal deoxyribonucleotidyl transferase and deoxyuridine triphosphate for 60 min. Nuclei were stained with DAPI (Invitrogen, USA). Cell apoptosis was evaluated by a fluorescence microscope (OLYMPUS, Japan) and calculated using Image-Pro Plus 6.0 software (Maryland, USA).

### Wound healing assay

HUVECs were grown up to 60–70% confluence in six-well plates. Then, cells were induced by H_2_O_2_ or/and treated with paeoniflorin or/and treated with EX527 and cultured at 37°C for 24 h. When the confluence was 100%, the cells were scratched by a 1000-μl disposable pipette tip and PBS was used to remove the dead cells. Images were taken by a digital light microscope (Olympus) at 0 h and 24 h after wounding.

### Tube formation assay

HUVECs were induced by H_2_O_2_ or/and treated with paeoniflorin or/and treated with EX527 and cultured at 37°C for 24 h. The 96-well plate was coated with Matrigel 30 min before this experiment. Next, HUVECs were seeded into the above 96-well plate (1 × 10^4^ cells per well) with serum-free M199 medium and incubated at 37°C. Images of the tube formation were obtained after 24 h with a light microscope (Olympus).

### Statistical analysis

All data were expressed as the mean ± standard deviation, and the statistical analysis was conducted using GraphPad Prism 8 (GraphPad Software, Inc.). Differences were calculated by Student’s t-test or one-way ANOVA followed by Turkey’s post hoc test. P < 0.05 was considered to indicate statistically significant differences.

## Results

### Paeoniflorin improves the pathological symptoms of gestational hypertension rats

The study analyzed L-NAME-induced gestational hypertension in rats by measuring mean arterial pressure (MAP), urine protein levels and histopathological sections. It was clear that significantly increased MAP in PIH rats was decreased after paeoniflorin treatment on D8 and D18 (Figure 1(a)). Urinary protein was markedly upregulated in the urine of PIH rats, which was reversed by paeoniflorin treatment on D9 and D19 (Figure 1(b)). H&E staining of rat placental tissue showed that in the PIH group, capillary density was remarkably smaller and the cytoplasm was looser compared to the control group. In contrast, the tissue status improved after paeoniflorin treatment and was extremely similar to the control group when paeoniflorin was administered at a dose of 300 mg/kg (Figure 1(c)).

**Figure 1.** Paeoniflorin improves the pathological symptoms of PIH rats. (a) The mean arterial pressure (MAP) in pregnant rats with or without Pae treatment was measured on day 8 and day 18 using a tail-artery pressure measuring instrument. (b) The urinary proteins in pregnant rats with or without Pae treatment was measured on day 9 and day 19 were detected by BCA method. (c) Histopathological damage of placenta tissue was observed by H&E staining. *P < 0.05, **P < 0.01 and ***P < 0.001.

### Paeoniflorin increases growth factor levels and decreases inflammatory factor levels in serum and placental tissues of gestational hypertension rats

Studies have analyzed growth factor levels and inflammatory factor levels by ELISA or Western blot, including PlGF, VEGF, sFlt-1, TNF-α, IL-6, IL-1β and MCP-1. In the serum of PIH rats, sFlt-1 level was increased while levels of PlGF and VEGF were decreased compared with control group, which were then reversed by paeoniflorin treatment in dose-dependent manner (Figure 2(a)). Similarly, in placental tissues of PIH rats, compared with control group, mRNA expression of sFlt-1 was enhanced while mRNA expressions of PlGF and VEGF were suppressed, which were subsequently reversed by paeoniflorin treatment in dose-dependent manner (Figure 2(b)). The results of Western blot analysis were consistent with that of RT-qPCR analysis in placental tissues (Figure 2(c)). As Figure 3(a) depicted, the enhanced levels of TNF-α, IL-6, IL-1β and MCP-1 in the serum of PIH rats were diminished after the treatment of paeoniflorin (Figure 3(a)). The changes of TNF-α, IL-6, IL-1β and MCP-1 contents in placental tissue of PIH rats in each group were consistent with that in serum (Figure 3(b)).

**Figure 2.** Paeoniflorin decreases the levels of sFlt-1, PlGF and VEGF in serum and placental tissues of PIH rats. (a) The levels of sFlt-1, PlGF and VEGF in serum of PIH rats with or without Pae treatment were determined by ELISA kits. The mRNA (b) and protein expressions (c) of sFlt-1, PlGF and VEGF in placental tissues of PIH rats with or without Pae treatment were detected by RT-qPCR and Western blot. *P < 0.05, **P < 0.01 and ***P < 0.001.

**Figure 3.** Paeoniflorin decreases the levels of inflammation in serum and placental tissues of PIH rats. The levels of TNF-α, IL-6, IL-1β and MCP-1 in serum (a) and placental tissues (b) of PIH rats with or without Pae treatment were determined by ELISA kits. *P < 0.05, **P < 0.01 and ***P < 0.001.

### Paeoniflorin decreases placental tissue oxidative stress level and increases serum nitric oxide (NO) level in gestational hypertension rats

The oxidative stress level in tissues and NO level in serum were analyzed by the corresponding kits, respectively. According to Figure 4, MDA level was upregulated in placental tissue of PIH rats, while the levels of SOD and GSH-Px were downregulated compared with control group, which were reversed by the treatment of paeoniflorin. It was noted that NO expression was reduced while iNOS expression was increased in the serum of PIH rats. In contrast, NO levels were increased and iNOS levels were suppressed after paeoniflorin treatment compared to the PIH group (Figure 5(a)). In addition, the low expression of eNOS in placental tissue in PIH group were increased by paeoniflorin treatment (Figure 5(b)). More importantly, SIRT1 protein expression in placental tissue of gestational hypertension rats increased by paeoniflorin treatment in dose-dependent manner (Figure 5(b)).

**Figure 4.** Paeoniflorin decreases the levels of oxidative stress in placental tissues of PIH rats. The levels of MDA, SOD and GSH-Px in placental tissues of PIH rats with or without Pae treatment were determined by ELISA kits. **P < 0.01 and ***P < 0.001.

**Figure 5.** Paeoniflorin promotes the expression of SIRT1, NO and eNOS and inhibits the production of iNOS in PIH rats. (a) The levels of NO and iNOS in serum of PIH rats with or without Pae treatment were determined by assay kits. (b) The expression of SIRT1 and eNOS in placental tissues of PIH rats with or without Pae treatment was analyzed by Western blot. ***P < 0.001.

### Paeoniflorin attenuated H_2_O_2_-induced HUVEC injury by upregulating SIRT1

To further explore the mechanism, the inhibition of SIRT1 by adding EX527 in H_2_O_2_-induced HUVEC was studied to investigate cell viability, apoptosis, migration, angiogenesis and NO levels, respectively. Different concentrations of paeoniflorin (50 μM, 100 μM and 200 μM) have no obvious effects on the viability of HUVECs (Figure 6(a)). The viability of HUVECs was decreased after H_2_O_2_ induction, which was then improved by paeoniflorin treatment. Notably, paeoniflorin with a dose of 200 μM exhibited the optimal promotive effects on cell viability (Figure 6(b)). SIRT1 expression was obviously downregulated in HUVECs after H_2_O_2_ induction. However, the decreased SIRT1 expression in H_2_O_2_-induced HUVECs was gradually enhanced with the concentration of paeoniflorin increases. Evidently, paeoniflorin exhibited promotive effects on SIRT1 expression in a dose-dependent manner and paeoniflorin with a dose of 200 μM had the optimal promotive effects (Figure 6(c)). Therefore, the concentration of paeoniflorin at 200 μM was selected for ensuing experiment. The apoptosis of HUVECs was increased after H_2_O_2_ induction. Paeoniflorin decreased the apoptosis of H_2_O_2_-induced HUVECs, which was reversed by EX527 treatment (Figure 6(d)). H_2_O_2_ induction suppressed the migration of HUVECs, which was reversed by paeoniflorin treatment. However, EX527 treatment partially abolished the promotive effects of paeoniflorin on migration in H_2_O_2_-induced HUVECs (Figure 6(e)). In a similar manner, tube formation was clearly disrupted after H_2_O_2_ induction compared to control, but increased after paeoniflorin treatment. However, the effect of paeoniflorin on tube formation was inhibited after EX527 treatment (Figure 6(f)). The expressions of NO and eNOS were downregulated in H_2_O_2_-induced HUVECs while iNOS expression was upregulated, which were reversed by treatment of paeoniflorin. The effect of paeoniflorin on the expressions of NO, eNOS and iNOS could be reversed by EX527 treatment (Figure 6(g-h)).

**Figure 6.** SIRT1 inhibition reverses the protective effects of paeoniflorin on endothelial dysfunction of H_2_O_2_-induced HUVECs. (a) The viability of HUVECs treated with different concentrations of Pae was observed by CCK-8 assay. (b) The viability of H_2_O_2_-induced HUVECs treated with different concentrations of Pae was observed by CCK-8 assay. (c) The expression of SIRT1 in H_2_O_2_-induced HUVECs treated with different concentrations of Pae was detected by Western blot. The apoptosis (d), migration (e) and tube formation (f) of H_2_O_2_-induced HUVECs treated with Pae and EX527 were respectively detected by Tunel assay, wound healing assay and tube formation assay. The expression levels of NO and iNOS were determined by assay kits (g) and protein expression of eNOS was analyzed by Western blot (h) in H_2_O_2_-induced HUVECs treated with Pae and EX527. *P < 0.05, **P < 0.01 and ***P < 0.001.

## Discussion

Paeoniflorin has a variety of pharmacological effects such as anti-inflammatory, anti-oxidation, anti-tumor, anti-apoptosis, neuroprotection and immune regulation [15–21]. Meanwhile, the safety of most antihypertensive drugs for fetuses lacks strict clinical trial verification, and animal experimental studies have found that some drugs will affect the growth and development of fetuses, which can seriously cause fetuses to be unsound [22]. A number of studies have found that endothelial dysfunction caused by various factors such as placenta, genetic factors, immune factors, maternal factors and oxidative stress have become the main research focuses [23]. In addition, endothelial vascular injury or dysfunction is an important factor affecting the occurrence of PIH which has close relation with sFlt-1, PlGF and VEGF [24]. More interestingly, previous studies have demonstrated that the inhibition of inflammation and oxidative stress can alleviate hypertensive symptoms in gestational hypertension rat models [25–27].

As one of the important angiogenesis factors, VEGF is involved in the formation of placental vascular network in early pregnancy, and it is of great significance to promote fetal growth and development in late pregnancy, which is mainly achieved by regulating the permeability of endodermal cells [28]. Lyall et al. [29] reported that with the aggravation of PIH, the synthesis and secretion of placental VEGF were significantly inhibited; meanwhile, the plasma content of VEGF was gradually decreased, further affecting the physiological function of vascular endothelial cells and trophoblast cells as well as aggravating placental ischemia and hypoxia. The expression of sFlt-1 (a member of the growth factor family) promotes the damage of placental vascular endothelial cells, leading to the occurrence of local inflammatory reaction, and improves the degree of placental vascular spasms [30]. Abnormal increase of sFlt-1 can promote the influx of calcium ion in smooth muscle cells of placental vessel wall and increase the concentration of intracellular calcium ions, thus promoting smooth muscle spasms and leading to the increase of placental perfusion resistance coefficient [31]. PlGF, which is mainly secreted by fuelingistrophic cells and vascular endothelial cells, is highly expressed in placental tissues. PLGF exhibited promotive effects on angiogenesis, proliferation, migration and invasion of trophoblast cells to regulate the function of trophoblast cells and the growth of placental blood vessels [32]. Here, we also observed that sFlt-1 expression was increased while expressions of PlGF and VEGF were decreased in serum and placental tissues of L-NAME-induced gestational hypertension rats. In addition, paeoniflorin alleviated the development of pregnancy hypertension in rats through downregulating sFlt-1 expression and upregulating the expressions of PlGF and VEGF in serum and placental tissues. Furthermore, the results of inflammatory factor assays in serum and placental tissues of L-NAME-induced gestational hypertension rats revealed that gestational hypertension promoted inflammation, whereas paeoniflorin inhibited inflammatory factor (TNF-α, IL-6, IL-1β and MCP-1) expression in a dose-dependent manner.

NO is a small molecule that plays an important role in the regulation of immunity and blood pressure and NO production in the body is affected by NOS [33]. Studies in a pregnant mouse model suggest that acute blockade of NOS inhibits NO synthesis, which leads to increased blood pressure and relieves the biological process of decreased vasoconstrictor response in the body. Inhibition of eNOS expression can lead to hypertension, proteinuria, thrombocytopenia, renal damage and fetal growth restriction [34,35]. The expression of iNOS in placental syncytiotrophoblast cells and umbilical cord endothelial cells was increased in gestational hypertension patients [36]. Notably, SIRT1 can activate the activity of eNOS through deacetylation, which in turn increases the production of NO, thus producing antioxidant and pro-endothelial-vasodilation effects [37]. In this study, expression levels of NO and iNOS in serum as well as SIRT1 and eNOS in placenta tissues of PIH rats were all changed as previous studies. Furthermore, in H2O2-induced HUVEC model, paeoniflorin promoted the NO and eNOS expressions and inhibits the production of iNOS, which could be partially reversed by EX527.

## Conclusion

Paeoniflorin attenuated vascular endothelial cell injury or dysfunction, inflammation and oxidative stress in gestational hypertension rats. This effect may be mediated through upregulation of SIRT1. The study also highlighted the therapeutic potential of paeoniflorin in the treatment of gestational hypertension.

## Data Availability

Data will be available on reasonable request.

## Highlights

1. Paeoniflorin improved the pathological symptoms of gestational hypertension in rats.
2. Paeoniflorin increased growth factor levels and decreased inflammatory and oxidative stress levels in gestational hypertensive rats.
3. Paeoniflorin attenuated H_2_O_2_-induced endothelial cell dysfunction by upregulating SIRT1.
